# *In Vitro* and *In Vivo* Neuroprotective Effects of Sarcosine

**DOI:** 10.1155/2022/5467498

**Published:** 2022-10-15

**Authors:** Arzugül Tanas, Özlem Özdemir Tozlu, Tuğba Gezmiş, Ahmet Hacimüftüoğlu, A. M. Abd El-Aty, Onur Ceylan, Adil Mardinoğlu, Hasan Türkez

**Affiliations:** ^1^Department of Molecular Biology and Genetics, Erzurum Technical University, Erzurum, Turkey; ^2^Department of Medical Pharmacology, Faculty of Medicine, Atatürk University, Erzurum, Turkey; ^3^Department of Medical Pathology, Faculty of Medicine, Atatürk University, Erzurum, Turkey; ^4^Science for Life Laboratory, KTH-Royal Institute of Technology, Stockholm SE-17121, Sweden; ^5^Centre for Host-Microbiome Interactions, Faculty of Dentistry, Oral & Craniofacial Sciences, King's College London, London SE1 9RT, UK; ^6^Department of Medical Biology, Faculty of Medicine, Atatürk University, Erzurum, Turkey

## Abstract

Alzheimer's disease (AD) is a neurodegenerative disorder characterized by behavioral and psychological symptoms in addition to cognitive impairment and loss of memory. The exact pathogenesis and genetic background of AD are unclear and there remains no effective treatment option. Sarcosine, an n-methyl derivative of glycine, showed a promising therapeutic strategy for some cognitive disorders. To our knowledge, the impacts of sarcosine supplementation against AD have not yet been elucidated. Therefore, we aimed to determine the neuroprotective potential of sarcosine in *in vitro* and *in vivo* AD model. *In vitro* studies have demonstrated that sarcosine increased the percentage of viable cells against aluminum induced neurotoxicity. In AlCl_3_-induced rat model of AD, the level of antioxidant capacity was significantly decreased and expression levels of *APP*, *BACE1*, *TNF-α*, *APH1A,* and *PSENEN* genes were elevated compared to the control group. Additionally, histopathological examinations of the hippocampus of AlCl_3_-induced rat brains showed the presence of neurofibrillary tangles (NFTs). However, the administration of sarcosine produced marked improvement and protection of AD-associated pathologies induced by AlCl_3_ in experimental rats. Therefore, this investigation may contribute to design novel therapeutic strategies using sarcosine for the management of AD pathologies.

## 1. Introduction

Alzheimer's disease (AD) is a progressive neurodegenerative disease characterized by loss of memory and cognitive functions [1]. AD is the most prevalent cause of dementia (account for 60-80% of all cases); around 47 million people worldwide are believed to be living with this disease [2]. The number of Alzheimer's patients is expected to double every 20 years, so it is expected to be 72.7 million in 2030 and 131.5 million in 2050 [3]. Nowadays, there is no effective medication for AD. However, there are available thereapies that can decrease or slow up some symptoms and improve quality of life. Since the first diagnosis of Alzheimer's disease, FDA has approved only 6 drugs such as cholinesterase inhibitors, NMDA receptor antagonists and amyloid beta-directed monoclonal antibodies [4–7].

In 1907, Alois Alzheimer described neurofibrillary tangles and amyloid plaques in the brain, which, together with neuronal dystrophy and vascular alterations, are dedicated to creating the quality of the disorder [8]. Although the cause of AD is not clearly understood, it is believed that both genetic and environmental factors may work in concert to cause the disease [9].

It is generally acknowledged that excessive amounts of amyloid-*β* (A*β*) in the brain of an individual is the most crucial factor involved in *the* pathogenesis of AD. A*β* is generated from amyloid precursor protein (APP) by cleaving in one of two alternate ways [10]. The APP can be cleaved by *α*-secretase enzyme releasing large soluble APPs fragments into the extracellular space. Then, the second cleavage is carried out by *γ*-secretase to yield a p3 fragment and AICD. Alternatively, cleavage of the APP may be processed by *β*-secretase (memapsin 2, BACE1) and subsequently by *γ*-secretase generating A*β* peptide and AICD [11]. Neurofibrillary tangles (NFTs) may eventually lead to AD. NFTs are composed of phosphorylated tau protein. Tau is a protein from the family of microtubule-assisted proteins (MAP) linked to chromosome 17. Tau protein is bound to microtubules and plays a vital role in stabilizing the microtubules, maintaining the integrity of the cytoskeleton, and axonal conduction. NFTs cause changes in cytoskeleton, axonal transport, and impaired neuronal function. At the end of a certain period, NFTs appear to be involved in neuronal dealth [12]. In the AD process, tau protein is highly phosphorylated, in turn its capacity to bind microtubules decreases. The unbound tau protein forms NFTs by collapsing into the cell as double-stranded fibers. Although there is a correlation between NFT density and the severity of dementia, there is still a debate about the exact role of tau in the pathogenesis of AD. It has to be noted that the normal localization of tau protein and its role in stabilizing microtubules suggest that its dysfunction in axons can substantially contribute to the development of AD. It has been previously shown that there is a link between amyloid fibrils and molecular signal cascade triggering tau hyperphosphorylations [13].

Oxidative stress is implicated in a number of neuropathological disorders, according to growing experimental evidence [14, 15]. Reactive oxygen species (ROS) production includes oxidative alterations in biomolecules such as lipids, proteins, and nucleic acids, which in turn degrade cellular function and ultimately result in neurodegeneration in the brain [16]. Another key mechanism through which the presence of A*β* induced oxidative stress is neuroinflammation. Neuroinflammation, which includes the abnormal activation of glial cells and the production of various proinflammatory cytokines, is an important part of A*β* pathogenesis [17]. After A*β* production, microglia initiate an innate immune response that contributes to neuronal damage and cognitive decline, leading to sustained production and secretion of proinflammatory mediators, including interleukin (IL)-6, IL-1*β*, and tumor necrosis factor-*α* (TNF-*α*) [18, 19].

Aluminum (Al) is one of the most widely used toxic metals and is currently used in many products. Although Al has no known function in the human body, it changes the regulation of various ions in the body and causes a change *in* protein/lipid structure and function [20, 21]. Extreme exposure to Al can cause accumulation in tissues such as the brain, bone, liver, kidneys, skeletal systems, immunological systems, and reproductive systems [22, 23]. The brain is one of the most affected tissues, as aluminum can enter the brain through the high-affinity transferrin receptors across the blood-brain barrier (BBB) [24].

Al accumulation might be associated with the etiology of various neurological disorders, such as dementia, senile dementia, and AD [25, 26]. In patients with AD, the two lesions-senile plaques and neurofibrillary tangles are found in aluminum, suggesting a causal association between Al exposure and AD [27]. Sarcosine, an N-methyl derivative of glycine, is a natural amino acid found in muscles and other body tissues. It is metabolized to glycine by glycine dehydrogenase enzyme (Figure 1). Sarcosine is a naturally occurring GlyT1 inhibitor that increases the concentration of glycine in the synaptic space and enhances NMDA receptor function [28]. It can lower the seizure threshold and thence may act as antipsychotics. Sarcosine causes the accumulation of glycine in synaptic cleft; in turn, can enhance neurotransmitter release at certain areas of the brain [29].

Based on this background, we aimed to determine the therapeutic potential of sarcosine, which is thought to have a neuroprotective effect in different AlCl_3_-induced AD models using a wide range of *in vitro* and *in vivo* parameters.

## 2. Materials and Methods

### 2.1. Cell Culture

The human SHSY-5Y cell lines were cultured in Dulbecco's modified Eagle medium (DMEM) (Gibco®, New York, USA) supplemented with 10% heat-inactivated fetal bovine serum (Gibco®, New York, USA), 1% penicillin and streptomycin, 1% L-glutamin in an incubator (37° C and 5% CO_2_, humidified atmosphere). For differentiation, the medium was replaced with DMEM: F12 containing fetal bovine serum (1% FBS) and 10 *μ*M retinoic acid (RA) (Sigma-Aldrich®, Milan, Italy). The media were renewed every 3 days with 1% FBS and 10 *μ*M RA containing medium. Cell differentiation was observed for 11 days with a light microscopy [30].

### 2.2. WST-8 Assay

Cell viability was measured using CVDK-8 (Ecotech Biotechnology Turkey) kit according to the manufacturer's manual. Briefly, 1 × 10^4^ − 1 × 10^5^ cells were seeded in 96-well plates and kept under appropriate culture conditions (37°C, 5% CO_2_) for 24 h to promote cell attachment. Afterward, cells were incubated with different concentrations (0-800 mg/L) of sarcosine and AlCl_3_ (200 mg/L) for 24 h. After incubation, CVDK-8 reagent was added to each well and incubated for 3 h. At the end of incubation period, the absorbance of each sample was measured at 450 nm in a microplate reader (Synergy-HT; BioTek Winooski, VT, USA). As a positive control, cells were treated with 0.1% (*w/v*) Triton X-100. Cell viability was calculated by using the following formula:

(1) $$\begin{array}{c} \%\cdot \text{Viable}\cdot \text{cell}=\left(\text{OD of experimental group}/\text{OD of control group}\right)\times 100. \end{array}$$

### 2.3. LDH Assay

LDH assay was performed using CytoSelect™ LDH Cytotoxicity Assay Kit (Cell BioLabs, San Diego, CA, USA) following the provider's instructions. Briefly, the cells were treated as mentioned above and at the end of the culture period; 90 *μ*L supernatant was transferred to a new plate to which 10 *μ*L reaction mixture was added to each well. The reaction was incubated for 30 min at room temperature in the dark. Eventually, the optical density was measured at wavelength of 450 nm in a microplate reader (Synergy-HT; BioTek Winooski, VT, USA). As a positive control, cells were treated with 0.1% (*w/v*) Triton X-100.

### 2.4. Metal Chelating Activity

An aliquot of sarcosine (200 *μ*mol/L) was aspirated to 48-well plates and then allowed to stand at room temperature for 30 min. Afterward, metals of CuSO_4_, AlCl_3_, FeCl_3_, and ZnCl_2_, each of 200 *μ*mol/L were added. Subsequently, the absorption spectrum of the sarcosine was measured wavelength ranges of 200-500 nm using the Biotek EPOCH spectrophotometer device.

### 2.5. Design of *In Vivo* Studies

Twenty-four female Sprague–Dawley rats (8 weeks old) weighing 250-300 g were used in the experimental work. Herein, the study was approved by Atatürk University Animal Experiments Local Ethics Committee (AÜHADYEK) (clearance no. 77040475-000-E.1800140631-1851). Animals were maintained at Atatürk University Experimental Research Center (ATADEM) as per the directions specified by CPCSEA guidelines. Rats housed in four groups in standard polypropylene cages were given food and water *ad libitum* and maintained in a temperature-controlled (25 ± 2°C) room with a *12* : *12* day/night cycle. The AD rat model was induced as described previously, with some modifications [31]. The rats were randomized into four groups (group A: control; group B: sarcosine; group C: AlCl_3_; group D: sarcosine + AlCl_3_). Animals in group A were fed on a normal diet without aluminium. In group B, animals were injected intraperitoneally with 3,6 mg/kg bwt/day whereas rats in group C were injected intraperitoneally with 5 mg Al/kg bwt/day for 28 consecutive days. In group D animals were administered sarcosine (3,6 mg/kg bw/day) and Al (5 mg Al/day/kg bw) by i.p for 28 consecutive days.

### 2.6. Haematological and Biochemical Analysis

Blood samples were taken from rats in all groups after decapitation. To obtain serum, blood samples were incubated for 40 min and centrifuged at 1500 g for 15 min. Serum samples were used to determine the level of several biochemical and haematological parameters. Biochemical and haematological analyzes were performed on an automatic analyzer using commercial biochemical reagent kits (Abris+, Russia) in accordance with manufacturer's recommendations [32].

### 2.7. Histopathological Examination

Brain tissues of treated and control rats were fixed in 10% buffered formalin solution in labeled bottles. Tissues were stained with Hematoxin-eosin (H-E) and examined under a standard light microscopy.

### 2.8. Total Oxidative Stress (TOS) and Total Antioxidant Capacity (TAC) Analysis

Total antioxidant capacity (TAC) assay and total oxidant status (TOS) assay were carried out to measure the antioxidative/oxidative capacity in brain tissue using commercially available TAC and TOS assay kits (Rel Assay Diagnostics®, Gaziantep, Turkey) [33].

### 2.9. *In Vivo* Micronucleus Assay

Smear slides were made from peripheral blood samples taken from each group of rat after treatment. Two slides per animal were prepared and air-dried. 24 h later, slides were fixed in absolute methanol for 10 min and stained with diluted Giemsa stain (10%) for 10 min using a modified Lazalde-Ramos ´s protocol. The MN in each sample was scored using manual microscopy (Zeiss) (100X), under immersion.

### 2.10. Total RNA Isolation, cDNA Synthesis, and PCR Array Studies

Total RNA was extracted from brain tissue using PureLink ™ RNA Mini Kit (Invitrogen, Stockholm, Sweden) according to the manufacturer's instructions. Total RNA was reverse transcribed to cDNA using “High Capacity cDNA Reverse Transcription Kit” (Applied Biosystems ™) according to the manufacturer's instructions. Quantitative real-time PCR was performed on a Real-Time PCR Detection System (Qiagen Rotor-Gene Q) using Sybr Green Master Mix (Applied Biosystems ™) according to the manufacturer's instructions. The primers used for RT-qPCR are listed in Table 1. The fold change in the expression of each gene was calculated using the ΔCt method [34].

### 2.11. Statistical Analysis

Statistical analysis was performed with SPSS® version 21.0. The results are given as mean ± standard deviation. One-way analysis of variance (ANOVA) was used for statistical evaluation and Duncan's test was used as post-hoc and the level of statistical significance was accepted as *p* < 0.05.

## 3. Results

### 3.1. Effect of Sarcosine on Aluminum-Induced Neurotoxicity in Differentiated SHSY-5Y Cells

WST-8 assay was performed to determine the toxicity of AlCl_3_ on differentiated SHSY-5Y cells. The results showed that AlCl_3_ caused concentration-dependent toxicity in cells (Table 1). The highest concentration of AlCl_3_ (800 *μ*M) decreased the viability of the cultures to 16.35%, whereas the lowest concentration (1.25 *μ*M) caused a cell death of 3.76% compared to the control group. To determine the neuroprotective effect of sarcosine in differentiated SHSY-5Y cells, different concentrations of sarcosine were treated with AlCl_3_-induced cells. Sarcosine was found to be safe at all tested concentrations (data not shown). Moreover, sarcosine treatment showed significant protective effect in ameliorating aluminum-induced cell death (Figure 1).

### 3.2. Metal Chelating Effect

The chelating potential of sarcosine in the presence of Al^+3^, Fe^+3^, Cu^+2^, and Zn^+2^ metals was monitored by UV-Vis spectrometry in the range of 200 to 500 nm. We found that the absorbance spectra of sarcosine had been significantly increased after the addition of Fe^+3^. (Figure 2).

### 3.3. *In Vivo* Studies

#### 3.3.1. General Effects

No deaths occured in any of the four groups during the 4-week treatment period. Rats exposed to AlCl_3_, sarcosine, or both of them, did not show significant differences in body weight gain in comparison with the respective control groups (data not shown). On the other hand, Al treatment caused significant reduction in the weight of the whole brain of rats compared with control. It has to be noted that there was no significant difference in the weight of the whole brain of rats in groups B and D.

#### 3.3.2. Haematological and Biochemical Results

The results of haematological analysis of rats in control and treated groups are given in Table 2. AlCl_3_ exposure significantly increased WBC and RDW-SD levels compared to control group. On the other hand, the administration of sarcosine did not have a significant effect on these hematological findings compared to control. Besides, sarcosine treatment significantly ameliorated increased WBC and RDW-SD levels caused by AlCl_3_ exposure.

The results of biochemical parameters of control and experimental groups of rats are presented in Table 3. AlCl_3_ leads to *a* significant reduction of creatine kinase (CK), magnesium (Mg), creatine and uric acid levels. There were no significant changes in biochemical parameters of rats exposed to sarcosine.

#### 3.3.3. Histological Observation

Microscopic examination of H&E-stained sections of brain in control group showed a normal structure whereas severe histological changes including NFTs were observed in group C. On the other hand, numbers of NFTs were decresed in tissue sections from group D (Figure 3).

#### 3.3.4. Effect of Sarcosine on Antioxidative/Oxidant Activity in the Brain

We assessed the antioxidative/oxidative alterations in the brain by measuring TAC and TOS levels (Table 4). The TAC level of AlCl_3_ treated group was reduced by 37% in comparison with the control group. On the other hand, sarcosine treatment did not modulate the decreased TAC level by AlCl_3_. While AlCl_3_ increased the TOS levels by 43% compared to the control group; sarcosine administration could not alleviate the AlCl_3_ induced oxidative stress.

#### 3.3.5. Micronucleus Findings

Table 5 shows the results of the MN assay. The frequencies of MN in rats exposed to AlCl_3_ were significantly increased compared with control group (*p* < 0.05). Moreover, sarcosine modulated the increased MNHEPs rates by AlCl_3_.

#### 3.3.6. Molecular Genetic Responses

The *in vivo* results of the present study have demonstrated the protective role of sarcosine against AlCl_3_ induced neurotoxicity. In order to explore the molecular mechanisms underlying this neuroprotective effect, the expression levels of 14 selected genes were investigated. Significant differences in the expression levels of APP, BACE1, TNF-*α*, APH1A, and PSENEN genes were observed in experimental group exposed to AlCl_3_ when compared with the control group (Figure 4).

## 4. Discussion

Many research studies have shown that AlCl_3_ exposure causes the formation of amyloid plaques that are thought to initiate the pathogenesis of AD. Therefore, chronic exposure to AlCl_3_ is often used as an experimental model of AD [35–38]. Since AlCl_3_ has very strong neurotoxic effects, the discovery of effective agents against AlCl_3_ has paid much attention [37, 39]. It has been reported that sarcosine has a neuroprotective effect. In particular, studies have shown that the glutamate system is implicated in the pathogenesis of schizophrenia [40–42] and the beneficial effects of sarcosine on glutamate metabolism in the hippocampus [43, 44]. It is also proposed that sarcosine can be used as a treatment option for epilepsy [29]. Furthermore, sarcosine can be beneficial for patients receiving atypical antipsychotic risperidone. Consistent with this, significant clinical effects have been reported in patients receiving high-dose glycine in addition to atypical antipsychotics, clozapine and olanzapine [45]. However, the effects of sarcosine in AD-related changes have not been observed in other *reports*. Accordingly, we considered it worthwhile to investigate the potential of sarcosine to function as a neuroprotectant in an animal model of experimental AD induced by AlCl_3_. The present study demonstrated for the first time that treatment with sarcosine alleviated AlCl_3-_ induced neurotoxicity *in vitro* and *in vivo* models.

Oxidative stress, which occured via an imbalance in reactive oxygen species (ROS) and antioxidative defense, is one of the mechanisms which play a key function in the pathogenesis of several neurodegenerative diseases including AD [46–48]. In the present study, while the level of TAS was increased, the level of TOS was decreased in the brain of AlCl_3_-induced Alzheimer's disease rats. It has been shown that sarcosine is an effective agent to reduce oxidative stress and may be used as a neuroprotective candidate for moderating brain impairment in rat models [49]. Many reports have revealed that regulation of oxidative stress is effective in restoring brain damage [50, 51]. In parallel with this information, we revealed here that sarcosine administration significantly alleviated the biochemical changes induced by AlCl_3_ to normal values.

The previous study demonstrated the connection between oxidative stress and inflammation. The evidence indicates that oxidative stress contributes to the pathogenesis of chronic inflammatory diseases. Oxidative stress-related damages, such as glycated products, oxidized proteins, and lipid peroxidation, frequently cause neuronal degeneration, which is most commonly reported in brain disorders [52].

Oxidative stress is a crucial factor that could affect the onset and pathological development of AD [53, 54]. Excessive free radical accumulation causes oxidative damage to biological macromolecules, which further damages neural tissue and impairs cognitive function [55]. Inflammation and cell death caused by ROS in the brain tissues can eventually lead to neurodegeneration and memory loss because they alter synaptic and nonsynaptic interactions between neurons [52]. Additionally, neurological alterations such as neurofibrillary tangles, neural apoptosis, amyloid deposits, and mitochondrial dysfunction are frequently influenced by oxidative stress, which has been linked to the pathological development of AD [54].

Iron homeostasis within neurons is maintained by transferrin and ferritin. In the AD brain, altered iron homeostasis has been reported. In addition to high iron concentration, amyloid plaques usually contain transferrin primarily found in oligodendrocytes. Furthermore, an abnormal ferritin distribution has also been reported in AD [56]. In light of this information, the amino acid sarcosine can act as “metal chelators”, i.e. chelate Fe^+3^ forming a complex that can be used as preventive strategies against nucleic acid oxidation. Growing evidence supports that inflammation can be seen in some pathological regions of the brain with AD and does so with the complexity of local peripheral inflammatory responses. The accumulation of degenerative tissue and highly insoluble abnormal materials create the classic stimulants of inflammation [57]. The increase in WBC levels is therefore believed to be a marker of chronic inflammation [58]. In our study, we have found that the total WBC count was significantly higher in AlCl_3_ treated group than the control group. Notably, treatment with sarcosine *s*ignificantly reduced the level of WBC. High RDW (also known as red cell distribution widths) values are linked to a deficiency of folate or vitamin B12. In some studies, vitamin B12 deficiency was found to be higher in patients with AD, other dementia, and cognitive deficits than in controls [59]. In addition, low serum folate levels are linked to an increased risk of *AD* occurrence. On the other hand, some studies have shown positive effect of folate treatment on memory problems [60, 61]. While high RDW levels are suggested to be a new biomarker of inflammation, it is thought that it may support the role of inflammation in the pathophysiology of AD [62]. As a result of our hematological findings, RDW-SD values were significantly increased in AlCl_3_-induced experimental AD group, whereas it was significantly decreased following sarcosine treatment. It has therefore been shown that sarcosine has a protective effect in the AD model by decreasing inflammation.

CK is found in cells and tissues that consume ATP rapidly, such as skeletal muscle, brain, photoreceptor cells of the retina, spermatozoa, and smooth muscle. It also acts as an energy supply for fast buffering and regeneration of ATP [63]. CK has been shown to correlate with brain activity and protect the cell from toxicity by reducing ATP levels during hypoxia or chemically induced mitochondrial dysfunction [64]. In the light of this information, we found that CK level (in the experimental AD model induced by AlCl_3_) was decreased compared to the control group; the finding which is supported with others [[65, 66]. Further to that, we observed that sarcosine administration showed a significant increase in CK level compared to the AD model group.

There is a complex pathophysiological link between brain and kidney damage [67]. Removal of toxic, water-soluble nitrogenous wastes (of protein and nucleotide metabolism) by urine excretion is very essential for normal brain function. Impaired renal function may produce more burden for AD brain. Previous studies have attempted to address this complex, interdependent pathophysiological link, and stated that chronic kidney disease is one of the risk factors possibly leading to dementia and cognitive impairment [68, 69]. Therefore, renal failure may be considered as emerging evidence for AD. In our study, creatinine and uric acid levels of AD model group showed a significant decrease compared to the control group. Therefore, it can be suggested that AlCl_3_ induced renal and liver damage. These findings are in line for what has been reported in the literature for AD and kidney injury [70, 71]. The group in which sarcosine was given did not show a significant difference at the level to correct this decrease.

As a result of our molecular genetic findings, an increase in APP gene expression (which is the main event in the pathogenesis of AD) and an increase in BACE1, APH1a, and *Psenen* genes associated with amyloidogenic pathway were observed in experimental group of AlCl_3_. While Al decreasing *β*-secretase and *γ*-secretase activities, it decreases *α*-secretase activity.

In AD and other neurodegenerative diseases, neuroinflammation may lead to the release of a number of different pro-inflammatory cytokines, which promotes the process of neurodegeneration [72, 73]. According to recent studies, TNF-*α* level is associated with memory and cognitive impairment indicates memory defect, which is a characteristic feature of AD pathophysiology [74, 75]. Therefore, the increase in the TNF*-α* gene in the experimental group with Al exposure corresponds to the AD model. In this study, TNF-*α* were ameliorated in sarcosine-treated rats, reflecting its antioxidant and anti-inflammatory effect, matching with previous studies [72, 76, 77].

According to our results, AlCl_3_ causes pathogenesis related to AD. In addition, sarcosine does not have a negative effect on the analyzed genes and on the contrary, it shows a significant neuroprotective effect following administration.

## 5. Conclusion

In conclusion, the role of glycine derivative, sarcosine, against aluminum chloride*-*induced neurotoxicity has been found to be protective. First, it has been shown that this amino acid has a neuroprotective effect *in vitro*. Then, it was first reported that there was no hematotoxic, nephrotoxic, and hepatotoxic effect in *in vivo* study. It has been shown that sarcosine reduces oxidative stress, and as a hematological, biochemical, and genetically inhibitory effect on neurodegeneration induced by AlCl_3_ as well as it has a positive effect on the inflammation process. Moreover, sarcosine did not induce any genotoxic and cytotoxic effect. Additionally, it may act as a metal chelation therapy, forming a complex that can be easily removed from the body. Herein, we may propose sarcosine as a novel agent for treatment of AD, however, further preclinical and clinical trials are needed to prove our assumption.

## Figures and Tables

**Figure 1:** Neuroprotective effects of sarcosine on cell viability of differentiated SH-SY5Y cells against AlCl_3_ toxicity.

**Figure 2:** The chelating potential of sarcosine.

**Figure 3:** Representative images of brain tissues from experimental groups. a: Control group; b: AlCl_3_ group; c: AlCl_3_ + Sarcosine group (NFTs are indicated by arrows.).

**Figure 4:** Effects of sarcosine on gene expression level.

**Table 1:** Cytotoxicity of AlCl_3_ in differentiated SH-SY5Y cells. (*p* < 0.05).

AlCl_3_ concentration (*μ*M)	Cell viability (%)
1.25	96.24 ± 4.23
2.5	92.12 ± 5.01
5	83.54 ± 7.24
10	76.21 ± 8.32
25	73.24 ± 6.58
50	64.36 ± 4.32
100	61.27 ± 8.47
200	53.02 ± 7.06
400	33.25 ± 7.39
800	16.35 ± 6.21
Control	100

**Table 2:** Effects of sarcosine on haematological parameters (Values are presented as mean ± S.D.; *n* = 4, means in the table followed by different letter are significantly different at the (*p* < 0.05) level).

Parameter	Control	AlCl_3_	Sarcosine	AlCl_3_ + sarcosine
WBC	3.93 ± 0.29^a^	6.32 ± 0.44^c^	3.90 ± 0.08^a^	5.82 ± 0.18^b^
RBC	5.52 ± 1.12^a^	6.82 ± 0.86^a^	5.71 ± 0.35^a^	6.53 ± 0.79^a^
HGB	10.60 ± 0.71^a^	12.63 ± 1.16^b^	10.87 ± 0.85^a^	12.52 ± 0.33^b^
HCT	46.45 ± 2.10^b^	39.56 ± 1.65^a^	45.75 ± 2.35^b^	41.72 ± 3.53^a^
MCH	21.50 ± 0.57^b^	17.55 ± 1.60^a^	18.35 ± 0.56^a^	17.04 ± 1.36^a^
MCV	61.25 ± 1.89^b^	56.11 ± 2.75^a^	59.77 ± 2.70^b^	54.50 ± 1.29^a^
MCHC	31.65 ± 0.75^a^	30.00 ± 1.92^a^	30.75 ± 0.57^a^	31.05 ± 0.47^a^
RDW-SD	29.12 ± 2.01^a^	48.83 ± 4.70^c^	32.25 ± 2.06^a^	41.37 ± 2.80^b^
RDW-CV	15.50 ± 0.57^a^	23.54 ± 2.31^b^	17.46 ± 1.04^a^	21.97 ± 1.32^b^

**Table 3:** Effects of sarcosine on biochemical parameters (Values are presented as mean ± S.D.; *n* = 4, means in the table followed by different letter are significantly different at the (*p* < 0.05) level).

Parameter	Control	AlCl_3_	Sarcosine	AlCl_3_ + sarcosine
CK	656.25 ± 65.74^c^	424.93 ± 50.73^a^	635.00 ± 65.44^c^	545.25 ± 21.07^b^
AST	256.25 ± 11.08^a^	263.00 ± 7.21^a^	255.00 ± 4.08^a^	262.00 ± 5.71^a^
ALT	76.25 ± 1.70^a^	85.50 ± 2.88^b^	77.50 ± 2.08^a^	79.00 ± 1.82^a^
LDH	438.75 ± 38.99^a^	699.66 ± 51.04^b^	480.00 ± 46.90^a^	656.00 ± 37.69^b^
Triglycerides	85.25 ± 5.18^a^	75.50 ± 8.11^a^	80.00 ± 4.39^a^	79.50 ± 5.50^a^
Cholesterol	77.25 ± 3.20^a^	74.66 ± 3.07^a^	75.50 ± 2.88^a^	76.25 ± 5.85^a^
Ca	10.75 ± 0.58^b^	9.70 ± 0.08^a^	9.87 ± 0.76^a^	9.68 ± 0.05^a^
P	8.27 ± 0.61^a^	7.81 ± 0.60^a^	7.95 ± 0.54^a^	7.82 ± 0.22^a^
Mg	3.08 ± 0.28^b^	2.30 ± 0.14^a^	2.31 ± 0.14^a^	2.30 ± 0.20^a^
Creatinine	0.41 ± 0.06^b^	0.25 ± 0.05^a^	0.33 ± 0.03^ab^	0.28 ± 0.08^a^
Uric acid	7.20 ± 0.81^b^	3.04 ± 0.91^a^	6.32 ± 0.22^b^	3.55 ± 0.36^a^
BUN	22.64 ± 1.96^a^	20.38 ± 0.70^a^	20.75 ± 2.02^a^	20.63 ± 1.54^a^

**Table 4:** Effects of sarcosine on TAC and TOS level (Values are presented as mean ± S.D.; *n* = 4, means in the table followed by different letter are significantly different at the (*p* < 0.05) level).

Experimental groups	TAC level (mmol Trolox E/L)	TOS level (mmol H_2_O_2_ E/L)
Control	2.23 ± 0.24^b^	2.38 ± 0.25^a^
AlCl_3_	1.40 ± 0.30^a^	2.93 ± 0.15^b^
Sarcosine	2.11 ± 0.08^b^	2.46 ± 0.12^a^
AlCl_3_ + sarcosine	1.67 ± 0.10^a^	2.80 ± 0.13^b^

**Table 5:** Effects of sarcosine on frequency of micronucleus (Values are presented as mean ± S.D.; *n* = 4, means in the table followed by different letter are significantly different at the (*p* < 0.05) level).

Experimental groups	The frequency of micronucleus (MnPKE/1000 PKE)
Control	13.62 ± 2.32^a^
AlCl_3_	26.85 ± 2.06^b^
Sarcosine	13.83 ± 2.35^a^
AlCl_3_ + sarcosine	23.86 ± 1.40^b^

## Data Availability

The authors confirm that the data supporting the findings of this study are available within the article.

## References

[1] Xia X., Jiang Q., McDermott J., Han J.-D. J. (2018). Aging and Alzheimer’s disease: comparison and associations from molecular to system level. *Aging Cell*.

[2] Götz J., Bodea L.-G., Goedert M. (2018). Rodent models for Alzheimer disease. *Nature Reviews. Neuroscience*.

[3] Prince M. J., Wimo A., Guerchet M. M., Ali G. C., Wu Y. T., Prina M. (2015). *World Alzheimer Report 2015-The Global Impact of Dementia: An analysis of prevalence, incidence, cost and trends*.

[4] Park J., Lee S. Y., Shon J. (2019). Adalimumab improves cognitive impairment, exerts neuroprotective effects and attenuates neuroinflammation in an A*β*_1-40_-injected mouse model of Alzheimer's disease. *Cytotherapy*.

[5] Du X., Wang X., Geng M. (2018). Alzheimer’s disease hypothesis and related therapies. *Translational Neurodegeneration*.

[6] Haake A., Nguyen K., Friedman L., Chakkamparambil B., Grossberg G. T. (2020). An update on the utility and safety of cholinesterase inhibitors for the treatment of Alzheimer’s disease. *Expert Opinion on Drug Safety*.

[7] Matsunaga S., Kishi T., Nomura I. (2018). The efficacy and safety of memantine for the treatment of Alzheimer’s disease. *Expert Opinion on Drug Safety*.

[8] De Strooper B., Karran E. (2016). The cellular phase of Alzheimer's disease. *Cell*.

[9] Bird T. D. (1993). *Alzheimer Disease Overview*.

[10] Ghosh A. K., Brindisi M., Tang J. (2012). Developing *β*-secretase inhibitors for treatment of Alzheimer’s disease. *Journal of Neurochemistry*.

[11] Esen S. (2010). Alzheimer hastalığı patofizyolojisi: deneysel ve genetik bulgular. *Turkish Journal of Geriatrics*.

[12] Brion J. P. (1998). Neurofibrillary tangles and Alzheimer’s disease. *European Neurology*.

[13] Adalbert R., Gilley J., Coleman M. P. (2007). A*β*, tau and ApoE4 in Alzheimer's disease: the axonal connection. *Trends in Molecular Medicine*.

[14] Amin F. U., Shah S. A., Kim M. O. (2017). Vanillic acid attenuates A*β*_1-42_-induced oxidative stress and cognitive impairment in mice. *Scientific Reports*.

[15] Coyle J. T., Puttfarcken P. (1993). Oxidative stress, glutamate, and neurodegenerative disorders. *Science*.

[16] Khan M. S., Ali T., Kim M. W., Jo M. H., Il Chung J., Kim M. O. (2019). Anthocyanins improve hippocampus-dependent memory function and prevent neurodegeneration via JNK/Akt/GSK3*β* signaling in LPS-treated adult mice. *Molecular Neurobiology*.

[17] Ganguly U., Kaur U., Chakrabarti S. S. (2021). Oxidative stress, neuroinflammation, and NADPH oxidase: implications in the pathogenesis and treatment of Alzheimer’s disease. *Oxidative Medicine and Cellular Longevity*.

[18] Frost G. R., Jonas L. A., Li Y.-M. (2019). Friend, foe or both? Immune activity in Alzheimer’s disease. *Frontiers in Aging Neuroscience*.

[19] Ashour N. H., El-Tanbouly D. M., El Sayed N. S., Khattab M. M. (2021). Roflumilast ameliorates cognitive deficits in a mouse model of amyloidogenesis and tauopathy: involvement of nitric oxide status, A*β* extrusion transporter ABCB1, and reversal by PKA inhibitor H89. *Progress in Neuro-Psychopharmacology & Biological Psychiatry*.

[20] Lin R., Chen X., Li W., Han Y., Liu P., Pi R. (2008). Exposure to metal ions regulates mRNA levels of APP and BACE1 in PC12 cells: blockage by curcumin. *Neuroscience Letters*.

[21] Kawahara M., Kato-Negishi M. (2011). Link between aluminum and the pathogenesis of Alzheimer’s disease: the integration of the aluminum and amyloid cascade hypotheses. *International Journal of Alzheimer's Disease*.

[22] Exley C. (2013). Human exposure to aluminium. *Environmental Science. Processes & Impacts*.

[23] Cheraghi E., Golkar A., Roshanaei K., Alani B. (2017). Aluminium-induced oxidative stress, apoptosis and alterations in testicular tissue and sperm quality in Wistar rats: ameliorative effects of curcumin. *International Journal of Fertility & Sterility*.

[24] Rizvi S. H. M., Parveen A., Ahmad I. (2016). Aluminum activates PERK-EIF2*α* signaling and inflammatory proteins in human neuroblastoma SH-SY5Y cells. *Biological Trace Element Research*.

[25] Turkez H., Geyikoglu F. (2011). The efficiacy of bismuth subnitrate against genotoxicity and oxidative stress induced by aluminum sulphate. *Toxicology and Industrial Health*.

[26] Türkez H., Enes Arslan M., Stefano A. D. I., Cacciatore I., Mardinoğlu A. (2020). Nonpharmacological treatment options for Alzheimer’s disease: from animal testing toclinical studies. *Turkish Journal of Zoology*.

[27] El-Rahman S. S. A. (2003). Neuropathology of aluminum toxicity in rats (glutamate and GABA impairment). *Pharmacological Research*.

[28] Lechner S. M. (2006). Glutamate-based therapeutic approaches: inhibitors of glycine transport. *Current Opinion in Pharmacology*.

[29] Socała K., Nieoczym D., Rundfeldt C., Wlaź P. (2010). Effects of sarcosine, a glycine transporter type 1 inhibitor, in two mouse seizure models. *Pharmacological Reports*.

[30] Marinelli L., Fornasari E., di Stefano A. (2019). Synthesis and biological evaluation of novel analogues of Gly-l-pro-l-Glu (GPE) as neuroprotective agents. *Bioorganic & Medicinal Chemistry Letters*.

[31] Chen C.-L., Chang K.-Y., Pan T.-M. (2016). _Monascus purpureus_ NTU 568 fermented product improves memory and learning ability in rats with aluminium-induced Alzheimer's disease. *Journal of Functional Foods*.

[32] Türkez H., Geyikoğlu F., Keleş M. S. (2005). Biochemical response to colloidal bismuth subcitrate: dose-time effect. *Biological Trace Element Research*.

[33] Turkez H., Togar B., Tatar A., Geyıkoglu F., Hacımuftuoglu A. (2014). Cytotoxic and cytogenetic effects of *α*-copaene on rat neuron and N2a neuroblastoma cell lines. *Biologia (Bratisl)*.

[34] Nóbrega F. R. D., Ozdemir O., Bezerra Filho C. D. S. M. (2019). NFBTA: A Potent Cytotoxic Agent against Glioblastoma. *Molecules*.

[35] Gómez M., Esparza J. L., Cabré M., García T., Domingo J. L. (2008). Aluminum exposure through the diet: metal levels in A*β*PP transgenic mice, a model for Alzheimer's disease. *Toxicology*.

[36] Garcia T., Esparza J., Nogués M. R., Romeu M., Domingo J., Gómez M. (2010). Oxidative stress status and RNA expression in hippocampus of an animal model of Alzheimer’s disease after chronic exposure to aluminum. *Hippocampus*.

[37] Aly H. F., Metwally F. M., Ahmed H. H. (2011). Neuroprotective effects of dehydroepiandrosterone (DHEA) in rat model of Alzheimer’s disease. *Acta Biochimica Polonica*.

[38] Xiao F., Li X. G., Zhang X. Y. (2011). Combined administration of D-galactose and aluminium induces Alzheimer-like lesions in brain. *Neuroscience Bulletin*.

[39] Sood P. K., Nahar U., Nehru B. (2012). Stress proteins and glial cell functions during chronic aluminium exposures: protective role of curcumin. *Neurochemical Research*.

[40] de Bartolomeis A., Sarappa C., Magara S., Iasevoli F. (2012). Targeting glutamate system for novel antipsychotic approaches: relevance for residual psychotic symptoms and treatment resistant schizophrenia. *European Journal of Pharmacology*.

[41] Tsai G., Coyle J. T. (2002). Glutamatergic mechanisms in schizophrenia. *Annual Review of Pharmacology and Toxicology*.

[42] Müller N. (2008). Inflammation and the glutamate system in schizophrenia: implications for therapeutic targets and drug development. *Expert Opinion on Therapeutic Targets*.

[43] Strzelecki D., Szyburska J., Rabe-Jabłońska J. (2014). Two grams of sarcosine in schizophrenia–is it too much? A potential role of glutamate-serotonin interaction. *Neuropsychiatric Disease and Treatment*.

[44] Strzelecki D., Podgórski M., Kałużyńska O. (2015). Supplementation of antipsychotic treatment with sarcosine - GlyT1 inhibitor - causes changes of glutamatergic ^1^NMR spectroscopy parameters in the left hippocampus in patients with stable schizophrenia. *Neuroscience Letters*.

[45] Lane H.-Y., Huang C. L., Wu P. L. (2006). Glycine transporter I inhibitor, N-methylglycine (sarcosine), added to clozapine for the treatment of schizophrenia. *Biological Psychiatry*.

[46] Lin M. T., Beal M. F. (2006). Mitochondrial dysfunction and oxidative stress in neurodegenerative diseases. *Nature*.

[47] Gella A., Durany N. (2009). Oxidative stress in Alzheimer disease. *Cell Adhesion & Migration*.

[48] Barnham K. J., Masters C. L., Bush A. I. (2004). Neurodegenerative diseases and oxidative stress. *Nature Reviews. Drug Discovery*.

[49] Pinto M. C. X., Mourão F. A. G., Binda N. S. (2012). Pharmacological induction of ischemic tolerance in hippocampal slices by sarcosine preconditioning. *Neurochemistry International*.

[50] Kaur C., Ling E.-A. (2008). Antioxidants and neuroprotection in the adult and developing central nervous system. *Current Medicinal Chemistry*.

[51] Pan J., Zhang Q., Zhang Y., Ouyang Z., Zheng Q., Zheng R. (2005). Oxidative stress in heroin administered mice and natural antioxidants protection. *Life Sciences*.

[52] Popa-Wagner A., Mitran S., Sivanesan S., Chang E., Buga A.-M. (2013). ROS and brain diseases: the good, the bad, and the ugly. *Oxidative Medicine and Cellular Longevity*.

[53] Wang X., Wang W., Li L., Perry G., Lee H. G., Zhu X. (2013). Oxidative stress and mitochondrial dysfunction in Alzheimer’s disease. *Biochimica et Biophysica Acta (BBA)-Molecular Basis of Disease*.

[54] Zhao Y., Zhao B. (2013). Oxidative stress and the pathogenesis of Alzheimer's disease. *Oxidative Medicine and Cellular Longevity*.

[55] Bertram L., Tanzi R. E. (2008). Thirty years of Alzheimer’s disease genetics: the implications of systematic meta-analyses. *Nature Reviews Neuroscience*.

[56] Honda K., Casadesus G., Petersen R. B., Perry G., Smith M. A. (2004). Oxidative stress and redox-active iron in Alzheimer’s disease. *Annals of the New York Academy of Sciences*.

[57] Akiyama H., Barger S., Barnum S. (2000). Inflammation and Alzheimer's disease. *Neurobiology of Aging*.

[58] Zenaro E., Pietronigro E., Bianca V. D. (2015). Neutrophils promote Alzheimer's disease-like pathology and cognitive decline via LFA-1 integrin. *Nature Medicine*.

[59] Rieder C. R., Fricke D., Wang H. X. (2001). Vitamin B(12) and folate in relation to the development of Alzheimer’s disease. *Neurology*.

[60] Fioravanti M., Ferrario E., Massaia M. (1998). Low folate levels in the cognitive decline of elderly patients and the efficacy of folate as a treatment for improving memory deficits. *Archives of Gerontology and Geriatrics*.

[61] La Rue A., Koehler K. M., Wayne S. J., Chiulli S. J., Haaland K. Y., Garry P. J. (1997). Nutritional status and cognitive functioning in a normally aging sample: a 6-y reassessment. *The American Journal of Clinical Nutrition*.

[62] Öztürk Z. A., Ünal A., Yiğiter R. (2013). Is increased red cell distribution width (RDW) indicating the inflammation in Alzheimer's disease (AD)?. *Archives of Gerontology and Geriatrics*.

[63] Wallimann T., Wyss M., Brdiczka D., Nicolay K., Eppenberger H. M. (1992). Intracellular compartmentation, structure and function of creatine kinase isoenzymes in tissues with high and fluctuating energy demands: the ‘phosphocreatine circuit’ for cellular energy homeostasis. *Biochemical Journal*.

[64] Holtzman D., Brown M., O’Gorman E., Allred E., Wallimann T. (1998). Brain ATP metabolism in hypoxia resistant mice fed guanidinopropionic acid. *Developmental Neuroscience*.

[65] Smith C. D., Carney J. M., Starke-Reed P. E. (1991). Excess brain protein oxidation and enzyme dysfunction in normal aging and in Alzheimer disease. *Proceedings of the National Academy of Sciences of the United States of America*.

[66] Pettegrew J. W., Panchalingam K., Klunk W. E., McClure R. J., Muenz L. R. (1994). Alterations of cerebral metabolism in probable Alzheimer's disease: a preliminary study. *Neurobiology of Aging*.

[67] Ulusu N. N. (2015). Glucose-6-phosphate dehydrogenase deficiency and Alzheimer's disease: partners in crime? The hypothesis. *Medical Hypotheses*.

[68] De Ferrari G. V., Inestrosa N. C. (2000). Wnt signaling function in Alzheimer’s disease. *Brain Research. Brain Research Reviews*.

[69] Yu J., Gattoni-Celli M., Zhu H. (2011). Vitamin D3-enriched diet correlates with a decrease of amyloid plaques in the brain of A*β*PP transgenic mice. *Journal of Alzheimer's Disease*.

[70] Etgen T. (2015). Kidney disease as a determinant of cognitive decline and dementia. *Alzheimer's Research & Therapy*.

[71] Zammit A. R., Katz M. J., Bitzer M., Lipton R. B. (2016). Cognitive impairment and dementia in older adults with chronic kidney disease: a review. *Alzheimer Disease and Associated Disorders*.

[72] Yang N., Liang Y., Yang P., Wang W., Zhang X., Wang J. (2016). TNF-*α* receptor antagonist attenuates isoflurane-induced cognitive impairment in aged rats. *Experimental and Therapeutic Medicine*.

[73] Leng F., Edison P. (2021). Neuroinflammation and microglial activation in Alzheimer disease: where do we go from here?. *Nature Reviews. Neurology*.

[74] Cheng X., Shen Y., Li R. (2014). Targeting TNF: a therapeutic strategy for Alzheimer's disease. *Drug Discovery Today*.

[75] Decourt B., Lahiri D. K., Sabbagh M. N. (2017). Targeting tumor necrosis factor alpha for Alzheimer’s disease. *Current Alzheimer Research*.

[76] Janelsins M. C., Mastrangelo M. A., Oddo S., LaFerla F. M., Federoff H. J., Bowers W. J. (2005). Early correlation of microglial activation with enhanced tumor necrosis factor-alpha and monocyte chemoattractant protein-1 expression specifically within the entorhinal cortex of triple transgenic Alzheimer’s disease mice. *Journal of Neuroinflammation*.

[77] Nampoothiri M., John J., Kumar N., Mudgal J., Nampurath G. K., Chamallamudi M. R. (2015). Modulatory role of simvastatin against aluminium chloride-induced behavioural and biochemical changes in rats. *Behavioural Neurology*.

